The article "Biomarkers Associated with Cognitive Impairment in Treated Cancer Patients: Potential Predisposition and Risk Factors" was published in 2017. Journal: Front Pharmacol.

# Biomarkers Associated with Cognitive Impairment in Treated Cancer Patients: Potential Predisposition and Risk Factors

**DOI:** 10.3389/fphar.2017.00138

**Published:** 2017-03-21

**Authors:** Hélène Castel, Angeline Denouel, Marie Lange, Marie-Christine Tonon, Martine Dubois, Florence Joly

**Affiliations:** ^1^Laboratory of Neuronal and Neuroendocrine Differentiation and Communication, Institut National de la Santé et de la Recherche Médicale, DC2N, Normandie UniversityRouen, France; ^2^Institute for Research and Innovation in BiomedicineRouen, France; ^3^Cancer and Cognition Platform, Ligue Nationale Contre le CancerCaen, France; ^4^Institut National de la Santé et de la Recherche Médicale, U1086Caen, France; ^5^Medical Oncology Department, Centre François BaclesseCaen, France; ^6^Medical Oncology, University Hospital CenterCaen, France

**Keywords:** cognitive disorders, biological markers, predictive factors, cancer, chemotherapy

## Abstract

**Purpose:** Cognitive impairment in cancer patients induced, at least in part, by treatment are frequently observed and likely have negative impacts on patient quality of life. Such cognitive dysfunctions can affect attention, executive functions, and memory and processing speed, can persist after treatment, and their exact causes remain unclear. The aim of this review was to create an inventory and analysis of clinical studies evaluating biological markers and risk factors for cognitive decline in cancer patients before, during, or after therapy. The ultimate objectives were to identify robust markers and to determine what further research is required to develop original biological markers to enable prevention or adapted treatment management of patients at risk.

**Method:** This review was guided by the PRISMA statement and included a search strategy focused on three components: “cognition disorders,” “predictive factors”/“biological markers,” and “neoplasms,” searched in PubMed since 2005, with exclusion criteria concerning brain tumors, brain therapy, and imaging or animal studies.

**Results:** Twenty-three studies meeting the criteria were analyzed. Potential associations/correlations were identified between cognitive impairments and specific circulating factors, cerebral spinal fluid constituents, and genetic polymorphisms at baseline, during, and at the end of treatment in cancer populations. The most significant results were associations between cognitive dysfunctions and genetic polymorphisms, including APOE-4 and COMT-Val; increased plasma levels of the pro-inflammatory cytokine, IL-6; anemia; and hemoglobin levels during chemotherapy. Plasma levels of specific hormones of the hypothalamo-pituitary-adrenal axis are also modified by treatment.

The article "Biomarkers Associated with Cognitive Impairment in Treated Cancer Patients: Potential Predisposition and Risk Factors" was published in 2017. Journal: Front Pharmacol.

**Discussion:** It is recognized in the field of cancer cognition that cancer and comorbidities, as well as chemotherapy and hormone therapy, can cause persistent cognitive dysfunction. A number of biological circulating factors and genetic polymorphisms, can predispose to the development of cognitive disorders. However, many predictive factors remain unproven and discordant findings are frequently reported, warranting additional clinical and preclinical longitudinal cohort studies, with goals of better characterization of potential biomarkers and identification of patient populations at risk and/or particularly deleterious treatments. Research should focus on prevention and personalized cancer management, to improve the daily lives, autonomy, and return to work of patients.

## Introduction

There have been improvements in the efficacy of cancer treatments, and also in the management of side effects and patient care over the last decade. However, cancer treatments, most often chemotherapy, may induce side effects on the bone marrow, heart, cardiac, or digestive system and often cause nausea, alopecia, or even cognitive impairments Ahles (2012). Chemotherapy can cross the blood brain barrier (BBB) and cause brain damage (Cheung et al., 2015; Wang et al., 2015), which could explain cognitive impairments, including of concentration, memory, executive functions, and processing speed, symptoms often referred to as “chemofog” or “chemobrain” (Vardy et al., 2008; Joly et al., 2015). These cognitive disorders can have major consequences on patient quality of life, return to work, or autonomy, and thus represent a major public health issue which requires investigation.

To identify and characterize subgroups of patients at risk of cognitive impairment induced by cancer and its treatment, and to adapt patient treatment, it is essential to discover biological factors mediating cognitive problems and/or risk factors, such as genetic polymorphisms, inflammatory indicators, or blood biomarkers (Kesler et al., 2013; Wang et al., 2015). Some biomarkers, that are either predictive of risk or produced in response to treatment or the cancer itself, can be relatively easily measured by blood sampling before, during, and after management of the cancer. Such biological predictive factors may also correlate with cerebral imaging, to provide information about brain structure and volume changes involved in cognitive impairment (Wang et al., 2015).

The objective of this review was to establish a summary of original articles published since 2005, including all biological predictive factors of cognitive changes in cancer patients, particularly after cancer treatment. Moreover, we discuss the limitations of these studies, concerning their different types, methods, results, and interpretation.

The article "Biomarkers Associated with Cognitive Impairment in Treated Cancer Patients: Potential Predisposition and Risk Factors" was published in 2017. Journal: Front Pharmacol.

## Methods used for information stratification

Articles were retrieved from PubMed using the following key words:

- MeSH terms: “cognition disorders,” “neurotoxicity syndromes,” “biological markers,” “prognosis,” “biological factors”
- PubMed terms: “predictive factors,” “cancer,” “chemobrain,” “chemofog,” “cognitive dysfunction,” “cognitive impairments”

This review was guided by the PRISMA statement and used a search strategy focused on three components: “cognition disorders,” “predictive factors”/”biological markers,” and “neoplasms,” searched in PubMed (with MeSH and PubMed terms). Original studies since 2005 were included, regardless of type (i.e., cross-sectional and longitudinal, randomized, and non-randomized, single center and multicenter). Selection was not based on cancer type; mainly acute lymphoblastic leukemia (ALL), acute myeloid leukemia (AML), myelodysplastic syndrome (MDS), breast, lung, prostate, and differentiated thyroid carcinoma were included; however, brain tumors and cancers involving brain metastasis were excluded, because of their mass effects and potential consequences of surgery/resection on the brain, which are likely to directly impact cognitive function (Table 1). Moreover, all types of cancer treatments were included, except encephalic radiotherapy, which can have direct effects on brain function, edema, and cognition (Table 1). Studies for which predictive factors were cerebral and/or imaging parameters (magnetic resonance imaging/hippocampal volume or metabolic activity) or that did not address one or more of the three components, cancer, cognition, or biological mechanisms, were also excluded, along with clinical, physiopathological, and psychological parameters. Only human studies were included, thus preclinical animal studies were not taken into account.

**Table 1:** **Main antitumor treatments and their mechanisms of action reported within the 23 selected publications that can be linked to modified biological factors and cognitive dysfunctions**.

**Cancer type**	**Treatment**	**Mechanisms of action**
Breast	Leuprolide	GnRH agonist: reduce estrogen levels by continuous (and not pulsate) infusion of a GnRH action mimic
	Tamoxifen	Adjuvant hormonal treatment: blockage of estrogenic receptors (ER) in early and advanced ER-positive breast cancers
	Exemestane	orally active aromatase^a^ inhibitor: irreversible blockade of estrogen production
	Anti-aromatases	Competition with aromatase which blocks estrogen synthesis (not indicated in cited publications)
	Doxorubicin	Antibiotic intercalating DNA agent, inhibitor of Topoisomerase II, and oxygen free radical producer leading to toxicity
	Cyclophosphamide	Bifunctional inhibitor of DNA transcription and replication leading to mitotic cell apoptosis
	Docetaxel	Cytotoxic properties *via* inhibition of the microtubule dynamic during mitosis
	5-FU	Inhibition of thymidylate synthase (inhibition of DNA synthesis)
	Vincristine	Stop tubulin polymerization and block cell during metaphase
	Methotrexate	Inhibition of folic acid (cytotoxic effect) through inhibition of mitochondrial metabolism
ALL^b^	Methotrexate	Inhibition of folic acid (cytotoxic effect) through inhibition of mitochondrial metabolism
	Cytarabine	Block DNA synthesis during cell division
mRCC^c^ or GIST^d^	Sunitinib	Inhibition of tyrosine kinase receptors involved in tumor growth
	Sorafenib	Kinase inhibitor which leads decrease of tumor cell proliferation
	VEGFR inhibitors	Angiogenesis inhibitor (stop tumor growth)
	Radiotherapy	Tumor cell apoptosis by DNA deterioration

a *Aromatase, enzyme responsible of the biosynthesis of estrogen*.

b *ALL, Acute lymphoblastic leukemia*.

c *mRCC, metastatic renal cancer carcinoma*.

d *GIST, Gastrointestinal solid tumor*.

The article "Biomarkers Associated with Cognitive Impairment in Treated Cancer Patients: Potential Predisposition and Risk Factors" was published in 2017. Journal: Front Pharmacol.

The first exclusion criterion, evaluated by reading abstracts, was the absence of at least one of the three domains, i.e., “cognition disorders,” “predictive factors,”/“biological markers,” and “neoplasms.” Between 2005 and 2015, 65 studies at least partly covered the topic under investigation. Other exclusion criteria, determined by reading entire papers, concerned studies of brain tumors or cranial radiotherapy, or the absence of clear data on cognition and/or biomarker levels. Of the initially selected 65 studies, 23 were finally included in the analysis (Figure 1). These studies aimed to evaluate and characterize changes in several biological factors predictive for cognitive alteration in cancer patients, often in association with treatment. Different domains of cognition were assessed by batteries of neuropsychological tests and self-reports of cognitive function. The biological factors covered in this review are summarized in Tables 2–**6**. Most often, blood and serum samples were analyzed as simple and rapid tests with potential to provide information about the risk of cancer patients developing cognitive issues, and to facilitate identification of optimal treatment regimens for specific patient populations.

**Figure 1:** **PRISMA statement diagram illustrating the process of report identification, information selection and final inclusion for the present overview**. The first exclusion criterion form the reading of the abstract, concerns the absence of the 3 combined domain, i.e., “cognition disorders,” “predictive Factor”/”biological markers” and “neoplasms.” The second exclusion criterion after reading of the entire papers, concerns brain tumors, cranial radiotherapy or the absence of clear data on cognition and/or biological marker dosage.

The article "Biomarkers Associated with Cognitive Impairment in Treated Cancer Patients: Potential Predisposition and Risk Factors" was published in 2017. Journal: Front Pharmacol.

**Table 2:** **Summary of methods and results from selected studies concerning inflammatory response**.

**Authors**	**Type of study**	**Age Mean ± (*SD* or range)**	**Cancer location (*n*)**	**Treatment type**	**Studied factors**	**Measurements**			**Results**	
						**Biological tests**	**Assessed cognitive domains**	**Time of assessment**	**Observed cognitive impairments**	**Association with studied predictive factors**
**INFLAMMATORY RESPONSE**										
Cheung et al., 2015	Multi-center prospective cohort	50.5 ± 8.4	Breast (*n* = 99)	Chemotherapy (anthracycline)	IL-1β, IL-2, IL-4, IL-6, IL-8, IL-10, GM-CSF, IFN-γ, TNF-α	Sensitive multiplex immunoassay (Venipuncture)	- Processing speed - Response speed - Memory - Attention (battery of tests) - + Self-report functioning	➢ T1: Before chemotherapy ➢ T2: 6 weeks ➢ T3: 12 weeks after initiation of chemotherapy	- Response speed performance (2.2% of patients) - Memory (13.2%) - Attention (7.3%) - Processing speed (2.2%) - Response speed (4.2%) + Self-perceived cognitive disturbances (29.3%)	↗ IL-1β: Poorer response speed performance ↗ IL-4: better response speed and less cognitive complaints ↗ IL-6: more severe cognitive complaints
Ganz et al., 2013	Prospective, cross-sectional at basal line, longitudinal and observational cohort	51.3 ± 7.8	Breast (patient-received CT^a^: *n* = 49; No CT patients: *n* = 44)	Radiotherapy Chemotherapy (FEC^c^ or AC-T^b^)	IL-6, IL-1, TNF-α RII, CRP	Sensitivity ELISA tests (Venipuncture)	- Psychomotor - Executive functions - Verbal learning and memory - Visual learning and memory - Visuo-spatial and motor speed (battery of tests) - Cognitive complaints	➢ T1: before therapy ➢ T2: 6 months later ➢ T3: 12 months later	Memory complaints	↗ TNF-RII: memory complaints
Ishikawa et al., 2012	Cross-sectional, case-control	63 (23–83)	Solid malignancies (various types: advanced, inoperable or recurrent) (Patients: *n* = 50 Healthy controls: *n* = 33)	Chemotherapy	IL-1β, IL-1Ra, IL-2, IL-4, IL-5, IL-6, IL-7, IL-8, IL-9, IL-10, IL-12, IL-13, IL-15, IL-17, basic FGF, eotaxin, G-CSF, GM-CSF, IFN-γ, IP10, MCP-1, MIP-1α, MIP-1β, PDGF-BB, RANTES, TNF-α, VEGF	Multiplex cytokine array system (Venipuncture)	Cognitive complaints (2 items of the EORTC QLQ-C30)	➢ After chemotherapy	Not specified	IL-6 and VEGF: negative correlation with subjective cognitive functioning
Janelsins et al., 2012	Stratified, randomized, double-blinded, and longitudinal	52.2 ± 10.2	Breast (AC/CAF^d^: *n* = 27 CMF^e^: *n* = 27)	Chemotherapy (AC/CAF or CMF)	IL-6, IL-8, MCP-1	Colorimetric ELISA kits (Venipuncture)	- Heavy-headed - Thoughts muddled - Difficulty thinking - Concentration and forgetful - Self-report functioning	➢ Prior to on-study chemotherapy cycle 2 ➢ After 2 consecutive chemotherapy cycles	All subjective domains (12-44% of patients)	- AC/CAF: No significant correlation between IL-6 or IL-8 and cognitive complaints. Significant correlation between MCP-1 and forgetfulness, difficulties with concentration and thinking. - CMF: No significant correlation
Kesler et al., 2013	Cross-sectional, case-control	54.6 ± 6.5	Breast (Case: *n* = 42 Healthy Control: *n* = 35)	Chemotherapy Number of regimens	IL-6, TNF-αs	Sandwich immunoassay (ELISA) (Venipuncture)	- Verbal memory - Learning - Global intelligence (battery of tests) - + Cognitive complaints	➢ Mean 4.8 ± 3.4 years off-therapy	Verbal memory (objective and subjective)	-↗ IL-6, ↗ TNF-α levels: ↗ Memory difficulties. In the breast cancer group, ↘ left hippocampal volume associated with ↗ TNF-α and ↘ IL-6, with a significant interaction between these two cytokines
Meyers et al., 2005	Longitudinal	60.2 (21–84)	Acute Myelogenous Leukemia (AML) or Myelodysplastic syndrome (MDS) (*n* = 54)	Chemotherapy: lipodaunocin plus Cytoxan or topotecan, plus or minus thalidomide	IL-1, IL-1RA, IL-6, IL-8, TNF-α, (+ Hb)	Standard enzyme-linked immunoabsorbant assays	- Attention, - Graphomotor speed - Verbal fluency - Visual-motor scanning speed - Executive functions - Fine motor dexterity - Memory (battery of tests)	➢ Before treatment ➢ and after 1 month of therapy	- Memory - Verbal fluency - Cognitive processing speed - Executive function and fine motor dexterity	↗ IL-6 level: ↘ executive function ↗ IL-8 level: ↗ memory performance
Mulder et al., 2014	Cross-sectional, case-control	60 (38-81) (+ TKI)	Metastatic renal cell cancer (mRCC) or Gastrointestinal stromal tumor (GIST) (VEGFR TKI group: *n* = 30, patient controls: *n* = 20, healthy controls: *n* = 30)	VEGFR TKI^f^ (Sunitinib or Sorafenib)	Testosterone, sex hormone binding globuline, estradiol, albumin, vitamin B12, thyroid function, CRP, ESR^g^, LDH^h^ Serum IL-1β, IL-2, IL-4, IL-5, IL-6, IL-8, IL-10, IL-12, TNF-α, TNF-β, IFN-γ	Specific ELISA (Venipuncture)	- Learning and memory - Attention and concentration - Executive functions (battery of tests) - + Self-report functioning	➢ Sunitinib or sorafenib for at least 8 weeks	- Learning and memory, and executive functions:Both patient groups significantly worse than healthy - Cognitive complaints > VEGFR TKI patients vs. healthy	- ↗ levels of ESR: ↘ scores learning, memory, attention, concentration and executive function - CRP and neutrophils: ↘ scores learning and memory (VEGFR TKI group). - Correlation between markers of systemic inflammation and worse cognitive performances - No correlation between serum IL-8 and cognitive functioning, or between free testosterone or estradiol and neuropsychological tests
Shibayama et al., 2014	Cross-sectional	47 ± 52 (+RT) 46.6 ± 6.2 (-RT)	Breast (Exposition to adjuvant RT with 25 CT: *n* = 51, Unexposed with 26 CT: *n* = 54)	Adjuvant regional RT	Plasma IL-6	Chemiluminescent enzyme immunoassay (Venipuncture)	- Attention/ concentration - Immediate verbal and visual memory - Delayed recall (battery of tests)	➢ 1 year after the initial therapy	- Delayed recall and immediate verbal memory in radiotherapy group	↘ delayed recall mediated by ↗ plasma IL-6 level

a *CT, Chemotherapy*.

b *AC-T, Cyclophosphamide, doxycycline plus taxane*.

c *FEC, Fluorouracil, cyclophosphamide plus taxane*.

d *AC/CAF: cyclophosphamide, or cyclophosphamide plus fluorouracil*.

e *CMF, cyclophosphamide, methotrexate and fluorouracil*.

f *VEGFR TKI, Vascular endothelial growth factor receptor tyrosine kinase inhibitors*.

g *ESR, Erythrocyte sedimentation rate*.

h *LDH, Lactate dehydrogenase*.

The article "Biomarkers Associated with Cognitive Impairment in Treated Cancer Patients: Potential Predisposition and Risk Factors" was published in 2017. Journal: Front Pharmacol.

## Biological markers and cognitive impairments in treated cancer patients

### Plasma biomarkers

#### Plasma inflammatory responses

The main cytokines analyzed in the reviewed studies were the pro-inflammatory triad, interleukin-6 (IL-6), tumor necrosis factor-alpha (TNF-α), and interleukin 1β (IL-1β). As IL-6 is an early mediator of inflammation and a key component of the acute phase response, it can also moderate inflammation by dampening TNF-α and IL-1β responses. Currently, the exact mechanisms involved in the inflammatory response during cancer therapy are not fully understood. Nevertheless, in cancer patients, circulating levels of cytokines were often increased and could be significant determinants of the alteration of particular cognitive functions after chemotherapy (Meyers et al., 2005; Ishikawa et al., 2012; Cheung et al., 2015). Based on the study by Ishikawa et al. (2012), it was difficult to conclusively link the observed cognitive issues with chemotherapy treatment since (i) cytokines, including IL-6, were measured in patient populations suffering from various types of advanced and inoperable or recurrent cancers and (ii) the delay between the end of the treatment and the time of the plasma assay was not stated. The study conducted by Meyers demonstrated that at baseline, higher IL-6 levels were associated with poorer executive functions, confirming that cancers are associated with high levels of circulating cytokines, connected with cognitive dysfunction, before chemotherapy. A longitudinal study by Cheung et al. (2015) established that higher concentrations of IL-1β and IL-6 were associated with more severe cognitive disturbance, and that increased IL-1β specifically was associated with poorer response speed performance during or just after the end of a chemotherapy treatment episode (Cheung et al., 2015; Table 2). In contrast, elevated IL-4 levels were linked to better response speed and fewer cognitive complaints in patients with breast cancer (Table 2), suggesting that maintenance of IL-4 levels during cancer care is likely to be neuroprotective (Cheung et al., 2015). Interestingly, breast cancer patients treated with chemotherapy had significantly elevated IL-6 and TNF-α levels after approximately 5 years off-therapy, compared with healthy controls, with an interaction between these two cytokines (Kesler et al., 2013). This study was particularly informative, since it correlated increased cytokine levels with diminished hippocampal volume, which is associated with verbal memory function. In agreement, an independent correlation between higher plasma IL-6 levels and deteriorated memory performance was described in breast cancer patients exposed to adjuvant local radiotherapy (Table 2; Shibayama et al., 2014). Together, these data suggest that cancer leads to increased plasma levels of selected pro-inflammatory cytokines, and that increased plasma IL-6 levels, likely resulting from chemotherapy or radiotherapy, may be a key systemic factor involved in, and/or predictive of, cognitive dysfunction (Table 2).

The article "Biomarkers Associated with Cognitive Impairment in Treated Cancer Patients: Potential Predisposition and Risk Factors" was published in 2017. Journal: Front Pharmacol.

Besides IL-6, which was described as marker of both cancer-associated and cancer treatment-induced inflammation, studies of other cytokines were less frequently reported. A longitudinal cross-sectional study, including baseline measurements, demonstrated changes in a number of pro-inflammatory cytokines; however, only levels of TNF receptor type-II (TNF-RII) were significantly higher in plasma from chemotherapy-treated patients compared with those who did not receive chemotherapy, with no differences observed in IL-1ra, IL-6, or C-reactive protein (CRP; Ganz et al., 2013). In detail, significant correlations between plasma TNF-RII and self-reported memory complaints, but not cognitive dysfunction evaluated by neuropsychological tests, was demonstrated at baseline (associated with relatively diminished brain metabolism). The study also demonstrated increased TNF-RII over time in patients who had received radiotherapy (first end point), different chemotherapy regimens (second end point), and then endocrine therapy (third endpoint; Table 2), leading them to hypothesize that fatigue and cognitive complaints may be caused by disturbances in TNF pathways (Ganz et al., 2013).

The article "Biomarkers Associated with Cognitive Impairment in Treated Cancer Patients: Potential Predisposition and Risk Factors" was published in 2017. Journal: Front Pharmacol.

In addition to cancer-related increases in circulating cytokine levels, data reported by Janelsins et al. (2012) support the idea that some cytokines may be specifically up-regulated in response to chemotherapy, and contribute to the development of cognitive difficulties. The study compared cytokine levels of IL-6, IL-8, and monocyte chemoattractant protein-1 (MCP-1) in patients receiving doxorubicin (Dox)-based cyclophosphamide/cyclophosphamide plus fluorouracil (AC/CAF) or Dox-based cyclophosphamide, methotrexate and fluorouracil (CMF) chemotherapy. The results demonstrated augmentation and diminution of cytokine levels in the AC/CAF and CMF groups, respectively, over time from baseline (prior to chemotherapy) and after two consecutive chemotherapy cycles, with a significant difference in levels of IL-6 between the two groups, suggesting that chemotherapy can induce specific cytokine changes. However, the study was under-powered and the time-points for blood sampling (before chemotherapy cycle) and cognitive evaluation (after chemotherapy cycle) did not match, hence it is difficult to conclusively evaluate the link between cytokine/chemokine changes and cognition, other than the reported negative correlation between MCP-1 and forgetfulness, difficulty with concentration, and thinking (subjective complaints, Table 2; Janelsins et al., 2012).

Circulating cytokines associated with cognitive impairment in cancer patients during the course of treatment, or in survivors after the end of treatment, represented the most measurable and measured factors, and studies converged to suggest that chemotherapy could dysregulate cytokine levels, which may interfere with brain functioning, leading to cognitive impairment (Ahles and Saykin, 2007). Indeed, some cytokines, including IL-6, IL-1β, and TNF-α, could have causal roles by crossing the BBB via active transporters (Cheung et al., 2015) and can interact with synapses (Wang et al., 2015), thereby leading to systemic communication between peripheral cytokines and the brain, rather than central cytokine production. This hypothesis is supported by a recent study by Hayslip et al. (2015), which proposed direct intravascular oxidative modification of plasma proteins by chemotherapy, leading to monocyte release of TNF-α which, by diffusing through the BBB, could then activate cascades of events potentially causing cognitive impairment (Hayslip et al., 2015). They demonstrated that the exogenous anti-oxidant, sodium-2-mercaptoethane sulfonate (mesna), present only in blood and urine, reduced plasma protein oxidation and TNF-α levels in patients receiving Dox-containing chemotherapy (Hayslip et al., 2015). Also, the observation that changes in plasma TNF-α levels were linked to reduced left hippocampal volume in cancer patients receiving chemotherapy (Kesler et al., 2013), suggests that cerebral apoptosis, or other cell death mechanisms, are likely responsible for altered verbal memory performance. Such cell death mechanisms could be counteracted by neutralization of circulating cytokines.

The article "Biomarkers Associated with Cognitive Impairment in Treated Cancer Patients: Potential Predisposition and Risk Factors" was published in 2017. Journal: Front Pharmacol.

Although this hypothesis raises interesting therapeutic options, other studies did not show any significant correlation between plasma cytokine levels and cognitive impairment with or without chemotherapy (Pomykala et al., 2013). In fact, co-variations between metabolism in selected brain regions and cytokines were detected by comparing values at baseline and 1 year after treatment completion in a group of patients who received chemotherapy (Pomykala et al., 2013). Overall, there is a clear difficulty in postulating a direct link between any particular cytokine that may be specifically up-regulated by a specific chemotherapy and responsible for a selected type of cognitive dysfunction. The observed discrepancies between studies may be due to differences in chemotherapy regimens, time periods between measurement of cytokine plasma levels and the end of chemotherapy, measurements of cytokine levels in serum or plasma, or the variable sensitivities of the methods used for measurement. Principal tests applied were the enzyme-linked immunosorbent assay (ELISA), including different variants such as the high sensitivity multiplex immunoassay (Ganz et al., 2013; Kesler et al., 2013; Pomykala et al., 2013; Cheung et al., 2015), or regular and high sensitivity kits (Ganz et al., 2013). Currently, the detailed mechanisms underlying cognitive changes remain unclear and future studies are required to obtain more data about the direct or indirect links between inflammatory responses and brain disorders associated with cancer therapy. It will be important to further consider the role of cytokines as predictive biomarkers for cognitive impairment in cancer and cancer-treated patients and to propose new cytokine inhibitors or antagonists as therapeutic options.

#### Non-inflammatory biomarkers in blood and serum samples

Since tumors can expand through development of angiogenic features and via release of angiogenetic factors, including vascular endothelial growth factor (VEGF), recently introduced targeted therapies include inhibitors of tyrosine kinase VEGF receptor (VEGFR TKI) and drugs targeting VEGF itself. As VEGF is also involved in neurogenesis and brain vascularization, it might be supposed that levels of VEGF could be linked to cognitive impairments (Table 3, Ishikawa et al., 2012). Accordingly, its levels were determined in a cross-sectional study of metastatic renal cancer (mRCC) patients treated with VEGFR TKI (8 week treatment period). The patients exhibited elevated erythrocyte sedimentation rates (ERS), CRP levels, and neutrophil counts, that were negatively correlated with learning, memory, attention, concentration, and executive functions (Mulder et al., 2014); however, no correlations were found with cytokine, hemoglobin (Hb), or electrolyte levels, leucocyte counts, or VEGF levels in blood samples. In a more recent longitudinal study, 30% of mRCC patients treated with anti-angiogenics were found to develop fatigue and cognitive disorders, while VEGF plasma levels measured at baseline, and 3 and 6 months from baseline, were associated with fatigue, but not with cognitive dysfunction (Joly et al., 2016). The impact of TKI, and of cancer itself, should be investigated further to clarify the exact effects of TKI on inflammatory responses and other circulating plasma markers, such as Hb, detrimental to cognitive performance.

The article "Biomarkers Associated with Cognitive Impairment in Treated Cancer Patients: Potential Predisposition and Risk Factors" was published in 2017. Journal: Front Pharmacol.

**Table 3:** **Summary of methods and results from selected studies concerning other factors in blood and serum samples**.

**Authors**	**Type of study**	**Age mean ± (*SD* or range)**	**Cancer location (*n*)**	**Treatment type**	**Studied factors**	**Measurements**			**Results**	
						**Biological tests**	**Assessed cognitive domains**	**Time of assessment**	**Observed cognitive impairments**	**Association with studied predictive factors**
**BLOOD AND SERUM SAMPLES**										
Fan et al., 2009	Non-randomized sub-study	53 to 50	Breast (Patients received hEPO: *n* = 45, Patients with standard care: *n* = 42)	Chemotherapy as adjuvant or neoadjuvant treatment	Hb	Blood tests	- Global efficiency (MMSE) - Verbal memory - + Self-report functioning	➢ After chemotherapy	No significant difference between groups	- No association between Hb and cognitive functioning. - Protective effect of hEPO against delayed cognitive dysfunction not shown
Iconomou et al., 2008	Prospective, single-center, non-randomized	58.9 ± 9.9	Solid malignancy (*n* = 50) Breast, colorectal, lung, genitourinary	Chemotherapy	Anemia, Hb hEPO	Hb levels (Venipuncture)	- Global efficiency: - Orientation - Recording - Attention - Calculation - Recall - Language - Copying (MMSE)	➢ T1 = baseline ➢ Study completion-T2 = week 12	No clinically significant alterations during hEPO treatment	Change of Hb not related with change of objective or subjective cognitive performance
Mancuso et al., 2006	Prospective, observational	76.6 ± 4.8	Lung (*n* = 42)	Chemotherapy	Anemia, Hb	Haemoglobin level	- Global efficiency - Orientation - Recording - Attention - Calculation - Recall - Language and copying (MMSE)	➢ Before chemotherapy (baseline) ➢ after each CT cycle	Not specified	↗ Hb: positive correlation with MMSE value
Massa et al., 2006	Longitudinal	71.4 (68–75)	Solid malignancy: Lung, oral cavity, ovary, breast, endometrial colon, stomach (Cancer patients with anemia related to cancer chemotherapy: *n* = 10)	Chemotherapy + rHuEPO	Hb level	Blood tests	- Global efficiency	➢ Prior to start chemotherapy ➢ After 4, 8 and 12 weeks of treatment	Better cognitive functions	↗ Hb levels: ↗ cognitive functioning assessed by MMSE after 4, 8 and 12 weeks of rHuEPO treatment
Natori et al., 2015	Cross-sectional	45.5 to 50	Breast (pNF-H positive: *n* = 18 pNF-H negative: *n* = 58)	Chemotherapy Many regimens	pNF-H level	ELISA (Venipuncture)	- Nonverbal - Intellectual capacity - Premorbid intellectual quotient (battery of tests) - + Self-report functioning	➢ Naïve ➢ Different cycles of chemotherapy 1, 3 or 7 cycles, ➢ Completed chemotherapy for at least 24 months	No difference among the patient groups	- ↗ serum pNF-H level but no association with cognitive deficits
Tan et al., 2013	Longitudinal	71 (59–89)	Prostate (*n* = 50)	Leuprolide	Plasma Aβ40 and Aβ42^a^	ELISA	- Global efficiency - ± verbal episodic memory	➢ Before the first leuprolide injection (baseline), ➢ At 2, 4 and 12 months	Better memory performance (practice effect)	No association between Plasma Aβ40 and Aβ42 levels and cognitive efficiency or memory functions

a *Aβ40 and Aβ42 : amyloid-β peptides 40 and 42*.

The article "Biomarkers Associated with Cognitive Impairment in Treated Cancer Patients: Potential Predisposition and Risk Factors" was published in 2017. Journal: Front Pharmacol.

Several studies investigating the contribution of chemotherapy-induced anemia to cognitive impairment in cancer patients suggested that changes in Hb were linked to the development of cognitive impairment during chemotherapy. This was stressed in the elderly cancer population studied by Mancuso et al. (2006), were Hb levels were associated with quality of life, functional capacity, mental decline, and depression, suggesting that maintenance of normal Hb levels is essential to prevent cognitive decline during chemotherapy. Low powered studies on treatments with specific therapies, such as recombinant human erythropoietin (rHuEPO), led to show improved Hb levels which were correlated with better cognitive function (Table 3; Mancuso et al., 2006; Massa et al., 2006). When rHuEPO is administered several times each week, it can compensate for cancer and chemotherapy-induced anemia after approximately 3 weeks of chemotherapy. In a larger cohort study, Iconomou et al. (2008) observed no significant changes in cognitive function in responders, exhibiting increased Hb levels after 12 weeks of rHuEPO treatment, despite improvement of physical function and diminished fatigue (Iconomou et al., 2008). In contrast, other studies using the same types of cognitive tests failed to detect evidence for a protective effect of erythropoietin (EPO) against delayed cognitive dysfunction (24 months from the end of the treatment) in groups of patients with breast cancer receiving chemotherapy (Fan et al., 2009; Table 3).

The article "Biomarkers Associated with Cognitive Impairment in Treated Cancer Patients: Potential Predisposition and Risk Factors" was published in 2017. Journal: Front Pharmacol.

Other systemic biological markers were also highlighted. A relationship between androgen receptors and amyloid precursors has been described (Takayama et al., 2009). Increased levels of amyloid-β40 (Aβ40), a marker associated with the Alzheimer disease, did not appear to be associated with cognitive mini-mental state examination (MMSE) scores after leuprolide treatment in prostate cancer patients (Tan et al., 2013). However, this study had some limitations, including a lack of evaluation of the ratio Aβ40/Aβ42 in plasma, indicating that the interesting hypothesis of a possible impact of cancer treatment on Aβ plasma levels and cognition deserves further investigation (Table 3).

Another candidate plasma marker for cognitive dysfunction following therapy-induced brain damage is axonal phosphorylated neurofilament subunit H (pNF-H), levels of which are increased in the blood of patients who have had acute brain ischemic stroke compared with controls, and are associated with the severity of the stroke (Singh et al., 2011; Andreano et al., 2012). Thus, Natori et al. (2015) considered that pNF-H would constitute an interesting systemic biomarker of neuronal lesions and measured its levels in the serum of breast cancer patients at baseline, after one to seven cycles of different chemotherapy regimens, and 1 month–1 year after the end of therapy. They established that pNF-H levels increased with the number of chemotherapy doses administered, but did not find any correlation with neuropsychological scores (Natori et al., 2015; Table 4). This suggests that measurement of serum pNF-H in chemotherapy-treated cancer patients, alongside the application of more sensitive batteries of cognitive tests, may be worthwhile to further evaluate pNF-H as a biomarker of neural axonal damage and cognitive impairment.

**Table 4:** **Summary of methods and results from selected studies concerning hormonal factors**.

**Authors**	**Type of study**	**Age mean ± (*SD* or range)**	**Cancer location (*n*)**	**Treatment type**	**Studied factors**	**Measurements**			**Results**	
						**Biological tests**	**Assessed cognitive domains**	**Time of assessment**	**Observed cognitive impairments**	**Association with studied predictive factors**
**HORMONAL FACTORS**										
Andreano et al., 2012	Longitudinal, Case-control	41.9 (27–49)	Breast (Case: *n* = 20 Natural cycling women Control: *n* = 20)	Lupron (Leuprolide)	Cortisol, estradiol, progesterone, glucocorticoids	Salivary ELISA for cortisol, estradiol and progesterone + physiological stressor	- Working memory - Verbal paired associate memory - Narrative recall (level of emotional arousal was considered) (battery of tests)	➢ After treatment for cases ➢ during the mid-luteal phase of menstrual cycles for controls	Narrative recall: delayed recall for emotional material	-↘ ovarian hormone levels - No difference of salivary cortisol level after stress -↘ glucocorticoid responsiveness: absence of enhancement of memory consolidation for emotional material in cases
Jenkins et al., 2005	Prospective, longitudinal, case-control	67.5 ± 4.7	Prostate (Case: *n* = 32 Control: *n* = 18)	Leuprolide	Free and bound testosterone, β-estradiol, sex hormone-binding globulin	Serum, Not specified	- Auditory/verbal memory - Visual memory, - Working memory and attention, - Processing speed - Vigilance - Intelligence	➢ Before drug treatment (Baseline T1) ➢ at 3 months before radiotherapy (T2) ➢ 9 months later (T3)	- Verbal - Visual spatial - Processing speed	↘ bioavailable testosterone, but no correlation with cognitive performance
Moon et al., 2014	, Cross-sectional, case-control	70.9 ± 5.0	Differentiated Thyroid Carcinoma (Case: *n* = 50 Control: *n* = 90)	TSH-suppressive therapy	Free T_4_ and TSH levels	RIA (Venipuncture)	- Verbal fluency - language - global cognitive function - memory - visuospatial function - attention - executive function	➢ After at least 5 years of TSH-suppressive treatment	° No difference between patient and control groups	↗ T_4_ level: ↗ global cognitive and visuospatial functions

The article "Biomarkers Associated with Cognitive Impairment in Treated Cancer Patients: Potential Predisposition and Risk Factors" was published in 2017. Journal: Front Pharmacol.

### Hormonal factors

Endocrine function, specifically gonadal and stress hormones, may also contribute to cognitive difficulties during cancer treatment. To date, the results of research into hormonal factors remain inconclusive, and studies are often related to patients receiving hormonal therapy. For example, significant reductions in free testosterone and β-estradiol levels were detected in prostate cancer patients after 3 months exposure to leuprolide, and some changes in spatial memory also were observed during treatment; however, there was no association between the changes in hormonal factors and those in cognition (Jenkins et al., 2005; Table 5). When therapy to suppress thyroid-stimulating hormone (TSH) was administered to patients with differentiated thyroid carcinoma, a positive correlation between free serum T_4_ levels and cognitive processing speed was detected (Moon et al., 2014), suggesting that exogenous T_4_ supplementation can improve cognitive function in this group of patients. In addition, given that gonadal hormonal levels can influence the hypothalamic-pituitary-adrenal axis (HPA), the cognitive and endocrine effects of the cortisol activating stressor, cold pressor stress (CPS), were tested in breast cancer patients previously treated with chemotherapy, and then receiving Lupron (Andreano et al., 2012). The glucocorticoid (cortisol) response to CPS was absent in the cancer patient group compared with controls, and delayed recall performance was also impaired in the individuals with cancer (Andreano et al., 2012). Thus, stress-induced cortisol favoring memory consolidation can be selectively altered in cancer patients. Other than this interesting study relating regulation of the HPA axis to cognitive impairment in cancer patients, there is little evidence to link the role of chemotherapy, stress, and/or cancer on circulating hormone levels and cognition.

**Table 5:** **Summary of methods and results from selected studies concerning genetic predictive factors**.

**Authors**	**Type of study**	**Age mean ± (*SD* or range)**	**Cancer location (*n*)**	**Treatment type**	**Studied factors**	**Measurements**			**Results**	
						**Biological tests**	**Assessed cognitive domains**	**Time of assessment**	**Observed cognitive impairments**	**Association with studied predictive factors**
**GENETIC PREDICTORS**										
Kamdar et al., 2011	Prospective cohort	4.4 ± 3.9 −12.1 ± 11.3	ALL (*n* = 62)	Methotrexate chemotherapy	6 Genotype polymorphisms (folate pathway: MTHFR^a^ 677C>T MTHFR 1298A>C SHMT^b^ 1420C>T MS^c^ 2759 A>G MTRR^d^ 66A>G TSER^e^2R/3R TSER3R/3R	Genotyping essay by PCR (Venipuncture)	- Attention - Processing speed - Verbal fluency - Visuo-spatial motor speed (battery of tests)	Years after end of therapy: 5.3± 4.4	Global cognitive functioning: 44.3% of patients	Combined effect of multiple folate pathway polymorphisms (MS and MTHFR): ↗cognitive disturbance probability (attention and processing speed)
Krull et al., 2013a	Cohort	7.0 ± 3.11	ALL (*n* = 243)	Chemotherapy (without prophylactic cranial irradiation)	Many genetic polymorphisms	Genotyping by PCR (Venipuncture)	- General intelligence - Processing speed - Working memory - Sustained attention - + cognitive complaints (assessed by parents)	2 years completion of consolidation therapy	Sustained attention and attention difficulties reported by parents	MS (/ MAOA^f^/ APOE^g^) polymorphisms: ↗ Cognitive disturbance probability (attentiveness and response speed)
Small et al., 2011	Cross-sectional, Case-control	56.93 ± 9.01 (RT) 51.22 ± 8.63 (CT)	Breast (RT: *n* = 58 CT: *n* = 72 Healthy Controls: *n* = 204)	Chemotherapy and radiotherapy	COMT^h^ Genotype COMT-Val COMT-Met	DNA collection by saliva and genotyping	- Overall cognition - Episodic memory - Attention - Complex cognition - Verbal fluency - Motor speed (battery of tests)	6 months after end of treatments	° COMT-Val+ carriers performed worse than COMT-Met homozygote carriers: Attention, verbal fluency and motor speed	COMT-Val homozygote: ↗ Cognitive disturbances probability

a *MTHFR: 5,10-methylenetetrahydrofolate reductase*.

b *SHMT: serine hydroxylmethyltransferase*.

c *MS: methionine synthase*.

d *MTRR: methionine synthase reductase*.

e *TSER: thymidylate synthase enhancer region*.

f *MAOA : Monoamine oxidase A*.

g *APOE: Apolipoprotein E*.

h *COMT: Catechol-O-Methyltransferase*.

The article "Biomarkers Associated with Cognitive Impairment in Treated Cancer Patients: Potential Predisposition and Risk Factors" was published in 2017. Journal: Front Pharmacol.

### Genetic factors

There is relative heterogeneity among cancer patients regarding (i) the various domains of cognition that can be affected, including working memory, executive functions, verbal memory, and processing speed; and (ii) the proportion of patients exhibiting long-term cognitive deficits, independent of fatigue or emotional disturbances. This has prompted medical researchers to investigate potential predisposing factors for the development of cognitive impairment during cancer and its treatment. Indeed, immune status, cancer diagnosis in the elderly, and/or a number of key genetic polymorphisms can predispose to cognitive changes (Ahles and Saykin, 2007; Mandelblatt et al., 2013; Janelsins et al., 2014). Should studies clearly demonstrate genetic predisposition, this could enable adaption of treatment to specific patient populations. Accordingly, recent studies have shown that genetic factors may be linked to cognitive impairments in cancer patients after therapy; for example, the gene encoding apolipoprotein E (APOE), located in chromosome 19, which functions in lipid transport and regulation of inflammation. APOE has three allelic variants (E2, E3, and E4), which include various combinations of two single nucleotide polymorphisms, rs7412 and rs429358. Chemotherapy-treated breast cancer patients carrying APOE-4 allele E4, a well-known risk factor for Alzheimer's disease (Ahles, 2012), have a higher risk of cognitive dysfunction during the course of cancer treatment (Mandelblatt et al., 2013). Consistent with these findings, Krull et al. analyzed various polymorphisms among childhood ALL survivors, and identified three that were associated with neurocognitive disorders, such as attentiveness, response speed, or parent-reported attention problems. In particular, an association between APOE-4 and attention deficit was described in survivors (Table 5). This study also identified associations between a single nucleotide polymorphism in the genes encoding methionine synthase (MS), which is responsible for the conversion of homocysteine to methionine, and monoamine oxidase A (MAOA), which catalyzes the deamination of amines such as dopamine, serotonin, or norepinephrine, and attention difficulties (Krull et al., 2013a).

The article "Biomarkers Associated with Cognitive Impairment in Treated Cancer Patients: Potential Predisposition and Risk Factors" was published in 2017. Journal: Front Pharmacol.

The key role of neurotransmitters as potential predisposing markers, is stressed by the other polymorphism commonly reported as linked to cognitive impairments, the Val158 Met encoding single-nucleotide polymorphism in catechol-O-methyltransferase (COMT), which catalyzes the metabolic breakdown of catecholamines through the methylation of dopamine and noradrenaline (Ahles and Saykin, 2007). In detail, codon 158 of COMT on chromosome 22q11, can encode for either a valine or a methionine residue (Small et al., 2011). The valine-containing variant protein exhibits elevated activity, leading to enhanced neurotransmitter degradation and consequent diminished neurotransmission (Table 5). This polymorphism predisposed a subgroup of patients with breast cancer to a higher risk of diminished cognitive performance, including attention, verbal fluency, and motor speed, evaluated 6 months after the end of chemotherapy (Small et al., 2011).

Other genetic polymorphisms also appear to be implicated in cognitive changes, such as those regulating folate pathways. Kamdar et al. (2011) investigated six different polymorphisms in genes involved in the folate pathway in childhood ALL survivors (Kamdar et al., 2011; Table 5), and described two genotypes in genes encoding 10-methylenetetrahydrofolate reductase and sphingomyelin (SM) as significantly correlated with general neurocognitive impairment (Kamdar et al., 2011).

### Biological factors in cerebrospinal fluid

When attempting to identify direct biological factors associated with cognitive alterations in cancer patients, variations in levels detected in cerebrospinal fluid (CSF) would be expected to provide better information about causal links with, or consequences of, treatment. Relationships between alterations in phospholipids, SM, and lysophosphatidylcholine (LPC) concentrations, as markers of white matter integrity, and some domains of cognitive function, were identified in children with ALL before and during long periods of chemotherapy (methotrexate administration over a period of years; Krull et al., 2013b). SM and LPC were shown to increase in CSF following chemotherapy induction and were associated with motor speed or visual working memory, and verbal working memory, respectively (Table 6; Krull et al., 2013b). These data indicate the occurrence of early cerebral neurochemical and neurocognitive alterations during chemotherapy, suggesting that, in addition to the effects of cancer itself, there is a direct and rapid impact of chemotherapy on the brain (white matter), and that brain imaging of the white matter may be beneficial during methotrexate administration. Methotrexate alters mitochondrial oxidative metabolism by inhibiting recycling of nicotinamide adenine dinucleotide, leading to accumulation of monounsaturated fatty acids. Thus, Moore et al. (2008) evaluated fatty acid levels (ratio between monounsaturated/saturated) in the CSF of patients with childhood ALL treated with methotrexate for more than 3 years (Moore et al., 2008). The number of intrathecal methotrexate doses received during the first year was significantly correlated with an increase in the stearic/oleic acid ratio, which was negatively correlated with decreased global intelligence and academic mathematics ability, while the palmitic/palmitoleic acid ratio was negatively correlated with global intelligence alone (Table 6; Moore et al., 2008). Hence, these two studies strongly support a specific deleterious impact of chemotherapy on beta-oxidation and fatty acid metabolism in the brain, suggesting that membrane and myelin defects may accompany cognitive dysfunction in some populations of cancer patients.

The article "Biomarkers Associated with Cognitive Impairment in Treated Cancer Patients: Potential Predisposition and Risk Factors" was published in 2017. Journal: Front Pharmacol.

**Table 6:** **Summary of methods and results from selected studies concerning cerebrospinal fluid**.

**Authors**	**Type of study**	**Age mean ± (*SD* or range)**	**Cancer location (*n*)**	**Treatment type**	**Studied factors**	**Measurements**			**Results**	
						**Biological tests**	**Assessed cognitive domains**	**Time of assessment**	**Observed cognitive impairments**	**Association with studied predictive factors**
**CEREBROSPINAL FLUID**										
Krull et al., 2013b	Longitudinal	7.0 ± 3.11	ALL (*n* = 76)	ChemotherapyMethotrexate	CSF phospholipids (PE^a^, PI^b^, PC^c^, SM^d^, LPC^e^)	Extraction and separation by chromatography (lumbar punctures)	- General cognitive abilities - Processing speed - Working memory - Visual-motor integration - Academic functions (battery of tests)	➢After completion of induction therapy (initial assessment) ➢Consolidation period:- one year after the initial assessment, - 2 years after - 3 years after	- Motor speed - Verbal and visual working memory - Motor speed	- Association between early variations in SM and motor speed and in LPC and verbal working memory; - Association between later elevation in SM with decline in visual working memory
Moore et al., 2008	Longitudinal	7.83 ± 2.87	ALL (*n* = 26 with 7 with low-risk, 13 with standard-risk and 6 with high-risk ALL)	Chemotherapy Methotrexate	CSF monounsaturated and saturated fatty acids: (palmitic, stearic, palmitoleic and oleic acids)	Gas chromatography	- General intelligence - Visual-motor skills - Academic abilities (battery of tests)	➢At diagnosis, prior treatments (fatty acids) ➢achieved remission (baseline) ➢1 year later (cognitive abilities)	- Global intelligence - Academic math abilities - Visual motor skills declines	-↗ ratio stearic/oleic acids: negative correlation with global intelligence and academic math abilities -↗ ratio palmitic/palmitoleic acids: negative correlation with global intelligence
Protas et al., 2009	Longitudinal	7.59 (range 2–16)	ALL (*n* = 38)	Chemotherapy Number of regimens	CSF Tau protein	ELISA	- Intelligence quotient (verbal performance) (battery of tests)	➢At diagnosis ➢after induction treatment ➢during consolidation ➢before maintenance therapy	Not specified	Tau protein level (at the initiation of maintenance therapy) negatively correlated with verbal abilities

a *PE, Phosphatidylethanolamine*.

b *PI, Phosphatidylinositol*.

c *PC, Phosphatidylcholine*.

d *SM, Sphingomyelin*.

e *LPC, Lysophosphatidylcholine*.

The article "Biomarkers Associated with Cognitive Impairment in Treated Cancer Patients: Potential Predisposition and Risk Factors" was published in 2017. Journal: Front Pharmacol.

CSF analysis can also provide inform about the microtubule-associated protein tau, whose CSF levels have already been associated with neurotoxicity and neurodegenerative pathologies. There is a significant increase in tau protein after induction and during consolidation, compared with at the time of diagnosis, in ALL patients. The level of tau measured before maintenance therapy was negatively correlated with verbal abilities (Protas et al., 2009), suggesting probable neural cell injury.

Overall, studies of patients with ALL receiving methotrexate-containing chemotherapy regimens for long periods demonstrate robust links between cognitive domains, such as working memory or verbal abilities, and modified CSF components, such as fatty acids, phospholipids, and even tau protein, which plays an important role in Alzheimer's disease (Table 6). Although the sampling method to obtain CSF by lumbar puncture is more invasive than blood tests, it appears to provide promising predictive biological information relating to cognitive function in cancer patients, which could be highly useful in various settings.

### Co-morbidities and limitations

It is important to consider clinical, physiopathological, and psychological factors in addition to biological markers, in relation to cognitive impairment of patients with cancer. In particular, to evaluate the contribution of co-morbidities and associated treatments, is essential to understand patient history and knowledge of these factors can help to predict cognitive impairments and determine the significance of changes in circulating factors in cancer patients during treatment. In support of this idea, in a study aiming to identify predictors of cognitive performance in breast cancer patients, treatment for hypertension was identified as having a significant negative impact on verbal fluency and working memory performance, and treatment for diabetes mellitus, was found to detrimentally affect executive functioning and reaction speed (Schilder et al., 2010). The same study also demonstrated that a higher number of “reproductive years” (as an indicator of lifetime estrogen exposure) appears to predict worse executive functioning. A longitudinal cohort study by Bender et al. (2013) demonstrated that before adjuvant chemotherapy, post-menopausal breast cancer patients exhibit poorer cognitive function than matched healthy controls; however, factors related to oral contraception were better predictors of verbal memory and attention in both controls and cancer patients (Bender et al., 2013), likely due to the positive biological impact of estrogen on brain function. The roles of various other factors, such as surgery, sleep disorders, anxiety, and cancer itself, on cognitive impairments specifically observed in cancer patients before chemotherapy, remain unknown. More generally, a study by Mandelblatt et al. (2014) revealed that elderly breast cancer patients with more advanced cancer or high levels of co-morbidity (including diabetes and cardiovascular disease) had higher rates of cognitive impairment than those with low co-morbidity levels, unlike matched control groups (Mandelblatt et al., 2014). These results highlight that some cancer patient populations are at risk of developing cognitive deficits as a result of cancer management, including chemotherapy.

The article "Biomarkers Associated with Cognitive Impairment in Treated Cancer Patients: Potential Predisposition and Risk Factors" was published in 2017. Journal: Front Pharmacol.

Several limitations should be noted in the studies analyzed in this report. There is an absence of meta-analyses, and the majority of available studies were prospective cross-sectional trials, mostly composed of small samples, and consequently had relatively low statistical power. Also, the studies included are not strictly comparable, because of the different methods used. Biological measurement methods are the main limit, and thus the variability in assessed cognitive domains and tests analyzed should also be considered in evaluation of this review. Indeed, some studies use global efficiency analyses, such as MMSE, whereas others applied batteries of tests, which are more sensitive for objective measurement of cognitive impairments. It should also be noted that practice effects can modify test results, particularly in longitudinal studies repeatedly using the same tests on patients after short periods of time. Finally, the large diversity of chemotherapy regimens used, inconsistent sampling points, and various cognitive assessment methods remain the major obstacles to identification of clear correlations between circulating biological factors levels and performance in specific domains of cognition. In addition, brain imaging could be an interesting approach to correlation of brain activity and biological markers in patients exhibiting no obvious cognitive impairment (Ferguson et al., 2007).

## Conclusion

A number of potential predictive markers have been identified that require validation in large series. Indeed, initial studies of factors, such as selected cytokines, stress hormones, CSF proteins, lipids, or Hb levels, have provided interesting information about changes in biomarkers that evolve during the course of the treatment of cancer patients, and also about genetic polymorphisms predisposing to cognitive deficits. Additional longitudinal studies, and investigation of other factors, previously identified in different pathological situations as associated with fatigue or aging, should facilitate better characterization of risk of cognitive impairment in cancer.

The question addressed in this study is among the priorities in cancer patient care and the ability to use biological risk factors to predict, better understand, and help to prevent cognitive issues, or adjust treatments for specific populations of patients identified as at risk, would be of major benefit. Such markers would also likely facilitate identification of biological mechanisms underlying neurotoxicity, and could open new avenues for testing and evaluation of therapeutic strategies designed to prevent cognitive dysfunction during cancer treatment, leading to improved quality of life, autonomy, and return to work rates of cancer survivors.

## Author contributions

HC and AD selected, read and analyzed articles. ML, MT, and MD built tables and analyzed cognitive domains evaluated in each study. HC and FJ supervised, organized and wrote the manuscript.

## Funding

Academic French governemental organization: Inserm and Normandie University, Anti-cancer center: Baclesse center, Caen, France

### Conflict of interest statement

The authors declare that the research was conducted in the absence of any commercial or financial relationships that could be construed as a potential conflict of interest.

## Abbreviations

AC/CAF: Cyclophosphamide/cyclophosphamide plus fluorouracil
ALL: Acute lymphoblastic leukemia
APOE: Apolipoprotein E
Aβ40 and Aβ42: amyloid-β peptides 40 and 42
CMF: Cyclophosphamide, methotrexate, and fluorouracil
COMT: Catechol-O-methyltransferase
CRP: C-reactive protein
CSF: Cerebrospinal fluid
CT: Chemotherapy
DNA: Deoxyribonucleic acid
Dox: Doxorubicin
ELISA: Enzyme-linked immunosorbent assay
EPO: Erythropoietin
GnRH: Gonadotropin-releasing hormone
Hb: Hemoglobin
IL: Interleukin
INFγ: Interferon γ
LPC: Lysophosphatidylcholine
MCP-1: Monocyte chemoattractant protein 1
MMSE: Mini-mental State Examination
MTHFR: 5,10-methylenetetrahydrofolate
mRCC: Metastatic renal cell cancer
pNF-H: Phosphorylated neurofilament subunit H
SM: Sphingomyelin
TNFα: Tumor necrosis factor-alpha
TNF-RII: Tumor necrosis factor-receptor type II
VEGF: Vascular endothelial growth factor
VEGFR TKI: Tyrosine kinase VEGF receptor
RT: Radiotherapy.
